The article "Gastroprotective Activity of Ethyl-4-[(3,5-di-tert-butyl-2-hydroxybenzylidene) Amino]benzoate against Ethanol-Induced Gastric Mucosal Ulcer in Rats" was retracted in 2023. Reasons: duplicated images; overlap with earlier publications; original data or images not available; unreliable data.

# Gastroprotective Activity of Ethyl-4-[(3,5-di-tert-butyl-2-hydroxybenzylidene) Amino]benzoate against Ethanol-Induced Gastric Mucosal Ulcer in Rats

**DOI:** 10.1371/journal.pone.0095908

**Published:** 2014-05-06

**Authors:** Mohammed Farouq Halabi, Raied Mustafa Shakir, Daleya Abdulaziz Bardi, Nahla Saeed Al-Wajeeh, Abdulwali Ablat, Pouya Hassandarvish, Maryam Hajrezaie, Anwar Norazit, Mahmood Ameen Abdulla

**Affiliations:** 1 Department of Biomedical Science, Faculty of Medicine, University of Malaya, Kuala Lumpur, Malaysia; 2 Department of Chemistry, Faculty of Science, University of Malaya, Kuala Lumpur, Malaysia; 3 Institute of Biological Science, Faculty of Science, University of Malaya, Kuala Lumpur, Malaysia; 4 Department of Medical Microbiology, Faculty of Medicine, University of Malaya, Kuala Lumpur, Malaysia; 5 Al-Moalim Mohamed Awad Center for Scientific Miracles of Prophetic Medicine, College of Medicine, Taibah University, Al-Madinah Al-Munawarah, Saudi Arabia; 6 Department. of Chemistry, Ibn Al-Haitham, University of Baghdad. Baghdad, Iraq; University of Valencia, Spain

## Abstract

**Background:**

The study was carried out to determine the cytotoxic, antioxidant and gastro-protective effect of ethyl-4-[(3,5-di-tert-butyl-2-hydroxybenzylid ene)amino] benzoate (ETHAB) in rats.

**Methodology/Principal Findings:**

The cytotoxic effect of ETHAB was assessed using a MTT cleavage assay on a WRL68 cell line, while its antioxidant activity was evaluated *in vitro*. In the anti-ulcer study, rats were divided into six groups. Group 1 and group 2 received 10% Tween 20 (vehicle). Group 3 received 20 mg/kg Omeprazole. Groups 4, 5 and 6 received ETHAB at doses of 5, 10, and 20 mg/kg, respectively. After an hour, group 1 received the vehicle. Groups 2–6 received absolute ethanol to induce gastric mucosal lesions. In the WRL68 cell line, an IC_50_ of more than 100 µg/mL was observed. ETHAB results showed antioxidant activity in the DPPH, FRAP, nitric oxide and metal chelating assays. There was no acute toxicity even at the highest dosage (1000 mg/kg). Microscopy showed that rats pretreated with ETHAB revealed protection of gastric mucosa as ascertained by significant increases in superoxide dismutase (SOD), pH level, mucus secretion, reduced gastric lesions, malondialdehyde (MDA) level and remarkable flattened gastric mucosa. Histologically, pretreatment with ETHAB resulted in comparatively better gastric protection, due to reduction of submucosal edema with leucocyte infiltration. PAS staining showed increased intensity in uptake of Alcian blue. In terms of immunohistochemistry, ETHAB showed down-expression of Bax proteins and over-expression of Hsp70 proteins.

The article "Gastroprotective Activity of Ethyl-4-[(3,5-di-tert-butyl-2-hydroxybenzylidene) Amino]benzoate against Ethanol-Induced Gastric Mucosal Ulcer in Rats" was retracted in 2023. Reasons: duplicated images; overlap with earlier publications; original data or images not available; unreliable data.

**Conclusion/Significance:**

The gastroprotective effect of ETHAB may be attributed to antioxidant activity, increased gastric wall mucus, pH level of gastric contents, SOD activity, decrease in MDA level, ulcer area, flattening of gastric mucosa, reduction of edema and leucocyte infiltration of the submucosal layer, increased PAS staining, up-regulation of Hsp70 protein and suppressed expression of Bax. *Key words*: ethyl 4-(3, 5-di-ter-butyl-2-hydroxybenzylamino) benzoate; toxicity; antioxidant; gastric-ulcer; anti-ulcer; histology; immunohistochemistry.

## Introduction

Schiff bases and their metal complexes containing the azomethine group derived from alkyl halogenated benzene are materials capable of electron-donating and electron-withdrawing activity [1]–[3], and they are widely employed as chelating agents especially in the field of coordination chemistry [4], [5]. The biological activities of such Schiff bases and their complexes are well known [4], [6]. They are reported to have antibiotic and anticancer activities [4], [7], [8]. In addition, they have been exploited industrially as fungicidal, and herbicidal agents [9]. Furthermore, their bio-efficacy on anti-tubercular and chelating potencies are reported to be remarkable [10]–[12].The potential *in vivo* bioactivity of these Schiff bases and their metal complexes are said to be due to the presence of O, N and S atoms, which interact *via* metal coordination with numerous bioactive metallo-biomolecules [4], [13]. In the literature, various bioactivities of synthetic chemical compounds including gastro-protective disorders have been reported [12], [14]–[16].

Gastric ulcer is one of the gastrointestinal disorders that have become a common global public health burden affecting a number of countries [17]. The etiology of the disease is reported to be due to the aggressive attack of different endogenous or exogenous factors on the alimentary canal's mucosal lining resulting in ulcerative lesions or excavations of gastric and duodenum tissue [18], [19]. Usually, the current approach in chemical drug management of gastric ulcer works through the inhibiting of gastric acid secretion or neutralization of the acid by antacid drugs, or the inhibiting of cellular apoptosis by the ‘cyto-protection’ effect resulting in an effective ulcer healing process [20], [21]. Although several types of chemical drugs are used in the treatment of gastric ulcer, unfortunately, most of them exhibit potent side effects such as arthralgia, arrhythmias, constipation, gynaecomastia, haemopoeitic changes, hypergastrinemia, hypocalcaemia, impotence and systemic alkalosis [19], [20].

In an effort to find novel alternatives to manage gastric ulcer, several newly synthesized chemical compounds are being investigated. Ethanol causes necrotic lesions that reduce gastrointestinal tract defensive factors like bicarbonate secretion and the production of mucus and its circulation [22]–[24]. In this study, we determine the cytotoxic, antioxidant and gastro-protective effect of ETHAB against ethanol-induced gastric mucosal ulcer in rats. We hope studies such as this will help to further highlight the reported bioactivities of these Schiff base complexes.

The article "Gastroprotective Activity of Ethyl-4-[(3,5-di-tert-butyl-2-hydroxybenzylidene) Amino]benzoate against Ethanol-Induced Gastric Mucosal Ulcer in Rats" was retracted in 2023. Reasons: duplicated images; overlap with earlier publications; original data or images not available; unreliable data.

## Materials and Methods

### Chemicals

#### ETHAB

The chemical compound (ETHAB) was synthesized according to Shakir et al. [1], and was provided by the Department of Chemistry, Faculty of Science, University Malaya, Malaysia. The crude was recrystallized from a hexane-ethanol mixture yielding a colorless crystal; yield 90% m.p. 137°C; IR.(KBr, U_max_ cm^−1^): 3480(br, OH), 3217 (br, NH), 1726(C = O), 1595, 1585 (C = C); ^1^HNMR (CDCl_3_, 400 MHz, ppm): 1.31(s, 9H, *o*-C(CH_3_)_3_), 1.38 (t, 3H, *J* = 7.1, OCH_2_ CH_3_), 1.42 (s, 9H, *p*-C(CH_3_)_3_), 4.21(s, 2H, CH_2_NH), 4.34(q, 2H, *J* = 7.2, OCH_2_), 4.46(bs, 1H, NH), 6.38(d, 2H, *J* = 8.8, H_9_), 7.05(d, 1H, *J* = 2.2, H_5_), 7.32(d, 1H, *J* = 2.4, H_3_), 7.35(bs, 1H, OH), 7.95(d, 2H, *J* = 8.8, H_10_);^13^CNMR (CDCl_3_, 100 MHz, ppm), 14.25 (1C,CH_3_), 29.60 (3C, *o*-C(CH_3_)_3_), 1.31.49(3C, *p*-C(CH_3_)_3_), 34.15(1C, *p*-C(CH_3_)_3_), 34.85(1C, *o*-C(CH_3_)_3_), 48.21(NHCH_2_), 60.47(OCH_2_), 114 (1C, C_11_), 121.91 (2C, C_9_), 124.12 (1C, C_3_), 124.16(1C, C_5_), 131.33(2C, C_10_), 136.65(1C, C_7_), 136.69(1C, C_2_), 142.18(1C, C_4_), 152.63 (1C, C_1_), 162.53(1C, CO). HREI/Ms. m/z = 383.2458 [M^+^] (calc. for C_24_H_33_NO_3_, 383.2460). ETHAB (Figure 1) was dissolved in 10% Tween 20 (Merck, Germany) as vehicle and was administrated orally in the experimental animal models.

**Figure 1:** Chemical structure of Schiff base ETHAB (ethyl-4-[(3,5-di-tert-butyl-2-hydroxybenzylidene)amino]benzoate).

#### Omeprazole

In this study, Omeprazole obtained from the University Malaya Medical Centre (UMMC) pharmacy, was used as the reference drug. The drug was dissolved in 10% Tween 20 and administrated orally at a dose of 20 mg/kg.

### MTT assay and cytotoxicity in cell line

Human liver embryonic cells, HeLa derivative (WRL68(was provided from department of molecular medicine, University Malaya. It was purchased from the American Type Culture Collection (ATCC, USA), and were used as a model cell line to evaluate the cytotoxic effect of ETHAB using a MTT assay (3-(4,5-dimethylthiazol-2-yl)2,5-diphenyl tetrazolium bromide) [25]. In brief, the cell line was cultured in RPMI-1640 growth medium, supplemented with ETHAB at different concentrations (3–100 µg/mL), 10% (v/v) sterile fetal bovine serum (FBS) (PAA Lab, Austria), 100 mg/mL streptomycin and 100 U/mL penicillin (PAA Lab, Austria) and 50 mg/mL fungizone (Sigma Aldrich). Cultures were incubated in a 5% CO_2_ incubator at 37°C in a humidified atmosphere. The cells were harvested by detaching the cells from the culture flask using trypsin after the flask reached confluency. MTT (5 mg) was added to 1 mL of phosphate buffer (pH 4.2) to give a MTT solution that was filter-sterilized. MTT solution (20 µL) was added to each well containing an equal volume of culture solution, and the micro-plates were further incubated at 37°C for 4 h with gyratory shaking. Supernatants were then discarded and 200 µL of acidified isopropanol (0.04 N HC1 in isopropanol) were added to the cultures and mixed thoroughly to dissolve the dark blue crystals of formazan. Thereafter, chromogenic formazan quantification was observed using an ELISA reader (TECAN, Mannedorf, Switzerland) at a 570 nm wavelength and a 690 nm reference wavelength [26].

The article "Gastroprotective Activity of Ethyl-4-[(3,5-di-tert-butyl-2-hydroxybenzylidene) Amino]benzoate against Ethanol-Induced Gastric Mucosal Ulcer in Rats" was retracted in 2023. Reasons: duplicated images; overlap with earlier publications; original data or images not available; unreliable data.

### Antioxidant property of the compound

#### DPPH free radical scavenging activity test

The antioxidant capacity of the compound to remove 1,1-diphenyl-2-picryl-hydrazyl radical was determined according to the method described by Shimada [27]. Briefly, in a 96-well plate, 30 µL of ETHAB in different concentrations (25–400 µg/mL) was added to 120 µL of freshly prepared 0.5 mM methanolic DPPH solution, mixed and kept in the dark for 20 min. The absorbance of the reaction mixture was read at 517 nm against a blank sample of methanol. The percentage of free radical scavenging activity was calculated according to equation (1):(1)where A1 is the absorbance of sample, and A2 is the absorbance of blank.

#### Ferric-reducing antioxidant power (FRAP) assay

The FRAP assay is based on the ferric reducing ability (antioxidant power) of plasma. The reducing ability is assayed based on the generated chromophore due to the reduction of ferric to ferrous ions resulting in the development of a blue colour complex [28]. The standard was tested at concentrations from 2.5 to 40 µg/mL. Ten (10) µL of the compound solution was mixed with 300 µL of the FRAP reagent in a 96-well microtiter-plate at 37°C, and incubated for 4 min. The mixture was then read spectrophotometrically using a microplate reader at 595 nm. The reducing concentration was ascertained using the absorbance of each sample against a standard curve obtained from iron (II) sulphate–heptahydrate (Fe_2_SO_4_. 7H_2_O).

#### Nitric oxide scavenging activity

The nitric oxide (NO) scavenging activity of the compound was evaluated using Griess reagent (Sigma, USA). The scavenging activity of all compounds was measured at different concentrations (25–400 µg/mL). Aliquot sample solution (50 µL) was mixed with 50 µL of sodium nitroferricyanide (10 mM) in phosphate buffered saline (PBS) (20 mM, pH 7.4) in a 96-well microplate. Thereafter, the mixture was incubated for 150 minutes followed by the addition of Griess reagent (125 µl). After 10 min, the absorbance was recorded at 546 nm with a microplate reader. Curcumin was used as the standard [29]. The percentage inhibition was calculated according to equation (2):(2)where A1 is the absorbance of control, and A2 is the absorbance of sample.

The article "Gastroprotective Activity of Ethyl-4-[(3,5-di-tert-butyl-2-hydroxybenzylidene) Amino]benzoate against Ethanol-Induced Gastric Mucosal Ulcer in Rats" was retracted in 2023. Reasons: duplicated images; overlap with earlier publications; original data or images not available; unreliable data.

#### Metal chelating assay

The metal chelating activity of the compound was evaluated according to a modified Wang et al. [30] protocol using different sample concentrations (25–400 µg/mL) and compared with the known standard ferrous ion chelator EDTA-Na_2_ (5–40 µg/mL). Sample solution (100 µl) was mixed with 135 µl of distilled water and 5 µl freshly prepared 2 mM FeCl_2_ solution in a 96-well microplate. Ferrozine (10 µL) was added to initiate the reactions. The mixture was then incubated for 10 minutes and the absorbance was read at 562 nm against water as the control, while the blank sample was without ferrozine. The metal chelating percentage was calculated according to equation (3):(3)where A0 is the absorbance of control, and A1 is the absorbance of compound or standard control (EDTA-Na_2_) and A2 is the absorbance of the blank sample. The concentration of compounds required to chelate 50% of the Fe^2+^ ions (IC_50_) was estimated from the graph against the percentage of inhibition.

### Experimental animals

#### Ethics statement

Animal work in this study was carried out in strict accordance with the United States Institute of Animal Research guidelines for the care and use of laboratory animals [31], and was approved by the Ethics Committee for Animal Experimentation, Faculty of Medicine, University of Malaya (Ethic No. PM/27/07/2012/HMF (R)). Throughout the experiment, all animals received humane care according to the regulations stated in the “Guide to the care and use of experimental animals” prepared by the Canadian Council for Animal Care [32]. Animals were sacrificed under anesthesia with ketamine/xylazine (0.5 mL of 100 mg/mL ketamine combine with 0.05 mL of 20 mg/mL xylazine) at a dosage of 0.55 mL/100 g body weight (b.w.).

#### Acute toxicity study

The acute toxicity of the compound was evaluated using thirty six (36) Imprinting Control Region (ICR) mice, 18 males and 18 females, with an average body weight of 25±4 g. The animals were assigned equally into 3 groups labeled as vehicle (10% Tween 20), low dose (500 mg/kg b.w.) and high dose (1000 mg/kg b.w.) of the compounds. Prior to administration, the animals were fasted overnight (food but not water) purposely to eliminate any food inside the gastrointestinal tract that might complicate absorption of the test substance. Food was withheld for a further 3 or 4 hours after dosing. The animals were observed at 30 min, 2, 4, 24 and 48 h after administration for the onset of clinical or toxicological symptoms as well as mortality and behavioral changes in the mice following the treatment. Mortality, if any, was observed over a period of 2 weeks. Animals were sacrificed on the 15^th^ day, and serum biochemical and histological (liver and kidney) parameters were determined following the standard method [33].

The article "Gastroprotective Activity of Ethyl-4-[(3,5-di-tert-butyl-2-hydroxybenzylidene) Amino]benzoate against Ethanol-Induced Gastric Mucosal Ulcer in Rats" was retracted in 2023. Reasons: duplicated images; overlap with earlier publications; original data or images not available; unreliable data.

#### Evaluation of compound's gastroprotective effect

In this analysis, thirty six (36) SD rats were used, divided equally into six (6) groups. The rats were fasted for 24 hours and singly housed in cages with a wide-mesh wire bottom to prevent coprophagy and dominancy. They were only allowed free access to drinking water, which was also removed three hours prior to the start of pretreatment. Animals were kept at room temperature (25°C) in humidity rooms on a standard light/dark cycle (12 h light/dark cycle). Samples were dissolved in 10% Tween 20 as vehicle, and administered orally via orogastric-intubations. Experimental gastric ulcer was induced according to the method described by Abdulla et al. [34] using ethanol as the model chemical for ulcer induction.

Group 1 (normal control), received 5 mL/kg b.w. of 10% Tween 20.

Group 2 (ulcer control) received 5 mL/kg b.w. of 10% Tween 20.

Group 3 (positive control) received 5 mL/kg b.w. of the standard drug Omeprazole (20 mg/kg).

Groups 4, 5 and 6 received 5 mL/kg b.w. of the compound at a dosage of 5, 10, and 20 mg/kg b.w., respectively.

After an hour, Group 1 received 5 mL/kg b.w. 10% Tween 20. Group 2–6 received 5 mL/kg b.w. absolute ethanol orally, and were humanely sacrificed under anesthesia an hour after administration. The pyloric and cardiac ends were tied and the stomachs were recovered for further tests.

#### Measurement of pH level and mucus weight

The removed stomachs were rapidly excised along the greater curvature, and the gastric juice was collected and centrifuged at 3000 rpm for 10 min. Collected mucus from each sample was analyzed based on mucus weight and pH (metric titration with 0.1 N NaOH solution). The stomach samples were then washed with iced PBS, and prepared for ulcer area measurement and homogenate as well as other histopathological examinations.

#### Macroscopical analysis of gross lesions

A dissecting microscope (1.8×) with a square-grid eyepiece was used to examine each gastric mucosa sample. The length (mm) and width (mm) of the ulcer on the gastric mucosa was measured using a planimeter (10×10 mm2). The area of each ulcer lesion was measured by counting the number of small squares, 2 mm×2 mm, covering the length and width of each ulcer band. The sum of the areas of all lesions for each stomach was applied in the calculation of the ulcer area whereby the sum of small squares ×4×1.8 =  ulcer area (mm^2^), as described elsewhere [16]. The inhibition percentage (I%) was calculated according to equation (4):(4)where A1 is the ulcer area of control, and A2 is the ulcer area of sample.

The article "Gastroprotective Activity of Ethyl-4-[(3,5-di-tert-butyl-2-hydroxybenzylidene) Amino]benzoate against Ethanol-Induced Gastric Mucosal Ulcer in Rats" was retracted in 2023. Reasons: duplicated images; overlap with earlier publications; original data or images not available; unreliable data.

#### Preparation for stomach homogenate

Gastric tissue was washed thoroughly with ice-cold saline. 10% (w/v) homogenate was prepared using Teflon homogenizer (Polytron, Heidolph RZR 1, Germany) in ice-cold 50 mM PBS (pH 7.4). The homogenate was centrifuged at 4,500 rpm for 15 min at 4°C [6]. The supernatant was used in evaluating the compound's antioxidant activity, total protein concentration, SOD and MDA level.

#### Evaluation of gastric total protein

The total protein in the stomach homogenate sample was evaluated based on the interaction between the higher molecular weight proteins and Coomassie Blue G250 dye. This interaction modifies the net charge of the dye molecule to change from cationic to anionic form. The gastric protein concentration was measured against an albumin standard curve. Samples were prepared according to Bradford [35]. In a micro-plate, 2 µL of the sample and 38 µL of the buffer solution were added to a well. Then, 200 µL of Bradford's solution that had been diluted (5×) was added to each well. After 5 min, the absorbance was recorded at a wavelength of 595 nm.

#### Measurement of antioxidant activity and membrane lipid peroxidation

The supernatant obtained from the stomach homogenate was used to assess SOD activity and MDA level following the manufacturer protocols for the commercial kits (Cayman, USA). The total protein concentration of each sample was determined using a Bradford assay [35].

#### Histological evaluation of gastric lesions

Samples from the gastric walls of each rat were fixed in buffered formalin (10%) and embedded in paraffin wax. These were then processed using a tissue-processing machine (Leica, Germany).

#### Hematoxylin and eosin staining

Sections of the stomach were made at a thickness of 5 µm, stained with hematoxylin and eosin (H&E), and thereafter analyzed microscopically following [36].

#### Study of mucosal glycoproteins

The mucosal glycoprotein changes were studied following the McManus method [37]. In this study, the glandular portion of the rat stomach was stained with Periodic Acid-Schiff (PAS), and the changes in the glycoproteins were compared.

The article "Gastroprotective Activity of Ethyl-4-[(3,5-di-tert-butyl-2-hydroxybenzylidene) Amino]benzoate against Ethanol-Induced Gastric Mucosal Ulcer in Rats" was retracted in 2023. Reasons: duplicated images; overlap with earlier publications; original data or images not available; unreliable data.

#### Immunohistochemical staining

Immunohistochemical staining was conducted according to the reported literature [12]. Commercial immunohistochemical reagents (Dakocytoma-tion, USA) were used. In brief, tissue section slides were heated at 60°C for approximately 25 min in a hot air oven (Venticell, MMM, Einrichtungen, Germany). The tissue sections were de-paraffinized in xylene and rehydrated using graded alcohol. Antigen was retrieved via microwave boiling of the sample in 10 mM sodium citrate buffer. Endogenous peroxidase was blocked using 0.03% hydrogen peroxide containing sodium azide. The tissue sections were washed gently with washing buffer, then incubated with Hsp70 (1∶500) or Bax (1∶200) biotinylated primary antibodies for 15 min. Thereafter, the sections were rinsed gently with washing buffer, placed in the buffer bath and kept in a humidified chamber.

The sections were then incubated with streptavidin–HRP (streptavidin conjugated to horseradish peroxidase in PBS containing an anti-microbial agent) for 15 min. After that, the tissue sections were rinsed gently in the washing buffer and placed in the buffer bath before being incubated with DAB-substrate-chromagenfor 5 min. The sections were then washed and counterstained with hematoxylin for 5 sec, then dipped in weak ammonia (0.037 M/L) 10 times and rinsed with distilled water prior to the mounting of the cover slips. Positive findings of the immunohistochemical staining were observed as a brown coloration in the tissue sections under a light microscope.

### Statistical analysis

Experimental data values were expressed as mean ± standard error mean (SEM). The statistical differences between groups were determined using statistical software (SPSS version 20). All obtained data were analyzed using Analysis of Variance (ANOVA) followed by post-hoc analysis. A probability value of *p<0.05* was considered as significant.

## Results and Discussion

### Evaluation of compound's cytotoxicity and acute toxicity

The MTT assay is one of the most commonly used colorimetric indices used to determine cytotoxicity and cell proliferation. The cytotoxic effect of Schiff base ETHAB was evaluated on the WRL68 cell line. The cells were treated with varying concentrations of the complex for 48 hours, and the viabilities were measured using the MTT assay. Our study revealed the compound to exhibit the ability to proliferate the viability of the WRL68 cell line (IC_50_>100 µg/mL) even at higher concentrations. This observation is further substantiated with the observed data from the acute toxicity analysis. The results of the current study showed that the LD_50_ of the compound was more than 1000 mg/kg with no appearance of any toxic behavior within the 14 days of the study. Furthermore, no significant changes or effects on the animal's clinical biochemistry test index in either sex were observed. This can be justified from the histological micrograph of liver (Figure 2, a–c) and kidney (Figure 2, d–f) samples. The histopathological evaluations of the sample sections revealed no detectable hepatic or renal toxicity and no appearance of any lesions or remarkable differences between the normal control and test groups. Based on this finding, it is therefore evident that oral administration of this compound up to 1000 mg/kg is safe. Similar observations on the absence of hepatic and renal toxicity in rats treated with Schiff base complexes at higher concentrations of up to 2000 mg/kg of body weight have been reported [6], [12], [14], [16], [24], [38].

The article "Gastroprotective Activity of Ethyl-4-[(3,5-di-tert-butyl-2-hydroxybenzylidene) Amino]benzoate against Ethanol-Induced Gastric Mucosal Ulcer in Rats" was retracted in 2023. Reasons: duplicated images; overlap with earlier publications; original data or images not available; unreliable data.

**Figure 2:** Histological study of acute toxicity in mice liver: (a) Mice orally administrated with 10% Tween 20 (normal group). (b) Mice orally administrated with low dose (500 mg/kg) ETHAB. (c) Mice orally administrated with high dose (1000 mg/kg) ETHAB. **Mice kidney**: (d) Mice orally administrated with 10% Tween 20 (normal group). (e) Mice orally administrated with low dose (500 mg/kg) ETHAB. (f) Mice orally administrated with high dose (1000 mg/kg) ETHAB. In all groups no lesions appear and no significant change compared to the normal control. (H&E staining, 20×).

### *In vitro* anti-oxidant tests

It has been reported that oxidative stress plays an important role in the pathogenesis of various diseases, including gastric ulcer [22]. The metabolic byproducts of ethanol are said to be comprised of superoxide anions and hydroperoxy free radicals that are implicated in the mechanism of acute and chronic ulceration in the stomach [39]. As such, antioxidant compounds are thought to ameliorate the damage caused by oxidative stress and, at the same time, to enhance the defense mechanism of the body. Several antioxidants have been reported to inhibit ethanol-induced gastric ulcer [38], [40]. In fact, Schiff bases are reported to play an important role in protecting against gastrointestinal diseases by acting as antioxidant and anti-inflammatory agents [41].

The results obtained from this study reveal the cytoprotective efficacy of ETHAB against gastric mucosa. For example, in the DPPH radical scavenging assay, the compound was observed to have an IC_50_ of 131.25±0.023 µg/mL in comparison to the observed BHA IC_50_ value of 5.9±0.01 µg/mL (Table 1). This was found to be in accord with Alam et al. [42], who studied the antioxidant activity of Schiff base 4-aminoantipyrine derivative and reported an IC_50_ value of 0.44 µM/mL, which was similar to their observed IC_50_ value of the standard drug, ascorbic acid (0.41 µM/mL). On FRAP evaluation, a value of 489.33±0.06 mmol Fe^2+^/mg compound was recorded for the compound. This corresponds to the observed IC_50_ 0f 141.20±0.02 µg/mL in NO and 73.1±0.12 in metal chelating assays (Table 1). The observed antioxidant activity of this compound could be the reason for its anti-ulcerogenic efficacy [14]. Indeed, Gwaram et al. [43] have illustrated the mechanism of Schiff base anti-oxidant cyto-protective activity to be through the presence of the carbonyl group (a well-known electrophilic acceptor) in the compounds, which appears to achieve antioxidant balance and to protect the gastric mucosa from injurious agents. Similar inhibition of NO by Schiff base 4-aminoantipyrine derivative has been reported [42]. The authors reported a significant reduction in NO production upon treatment with their synthesized Schiff base derivative. Similar studies have reported an observed significant increase in NO level upon pretreatment with dichlorido-zinc (II) Schiff base [13] and dichlorido-copper (II) Schiff base complexes [44].

The article "Gastroprotective Activity of Ethyl-4-[(3,5-di-tert-butyl-2-hydroxybenzylidene) Amino]benzoate against Ethanol-Induced Gastric Mucosal Ulcer in Rats" was retracted in 2023. Reasons: duplicated images; overlap with earlier publications; original data or images not available; unreliable data.

**Table 1:** IC_50_ values based on antioxidant evaluation of ETHAB in relation to other standard compounds.

Sample	DPPH IC_50_ (µg/mL)	FRAP mmolFe2+/mg compound	nitric oxide IC_50_ (µg/mL)	Metal Chelating IC_50_ (µg/mL)
**ETHAB**	131.25±0.023	489.33±0.06	141.20±0.02	73.12±0.12
**BHA**	5.95±0.01	-	-	-
**EDTA-Na**	-	-	-	8.96±0.03
**Curcumin**	-	-	1.54±0.07	-

All values are expressed as mean ± SEM.

### Evaluation of gastric ulcer parameters

#### Measurement of gastric contents pH and mucus weight

Mucus is an important factor in protecting the lining of the gastrointestinal tract. The gel mixture of water and glycogens that make up the mucus is reported to provide a kind of protective barrier against acidic aggressive attacks on the lining of gastrointestinal tract [44]. The obtained gastric contents was measured for pH and mucosal weight (M.W). The average readings are presented in Figure 3a and 3b. As expected, orogastric supplementation of ethanol in the ulcer control group (UC) significantly (*p<0.05*) reduced the pH (2.24±0.22) and mucus weight (180±40 mg) of the gastric contents resulting in high acidic conditions. On the other hand, in the other groups, pretreatment with ETHAB (5–20 mg/kg) or Omeprazole (PC) was found to significantly (*p<0.05*) restore the stomach pH and elevate the weight of mucus contents to the level observed in the normal control (NC) group (pH = 5.39±0.31 and M.W = 550±80 mg). In fact, pretreatment with ETHAB significantly (*p<0.05*) elevated the level of both pH and mucus weight in a concentration dependent fashion (Figure 3a & 3b). Pretreatment with 5 mg/kg ETHAB raised the gastric contents average pH to 3.97±0.39, while the average mucus contents was raised to 440±80 mg (Figure 3a & 3b). Increasing the ETHAB pretreatment concentration to 20 mg/kg resulted in a significant (*p<0.05*) increase in gastric contents pH (5.30±0.50) and mucus weight (540±50 mg), a level that is significantly (*p<0.05*) similar to that of both the normal and positive control groups (Figure 3a & 3b).The increase in mucus secretion in the pretreated group could be one of the factors that protected the newly formed gastric lining cells from further ethanol-induced gastric injury. Similar reports on the enhancement of mucosal secretion resulting in gastro-protection against ethanol-induced gastric ulcer by Schiff base copper II complexes have been recorded [44]. Furthermore, our observation concurs with Golbabapour et al. [6] who reported an increase in mucus weight upon treatment with Zinc II Schiff base derivative complex in acute supercritical hemorrhagic mucosal lesions in rats.

The article "Gastroprotective Activity of Ethyl-4-[(3,5-di-tert-butyl-2-hydroxybenzylidene) Amino]benzoate against Ethanol-Induced Gastric Mucosal Ulcer in Rats" was retracted in 2023. Reasons: duplicated images; overlap with earlier publications; original data or images not available; unreliable data.

**Figure 3:** (a) Effect of pretreatment with ETHAB on gastric contents pH. (b) Effect of pretreatment with ETHAB on mucus weight. (c) Effect of treatment with ETHAB on the ulcer area (mm^2^) and ulcer inhibition (%); number rat 6/group; *p<0.05*. All results are presented as average mean ± SEM. *The mean difference is significant at the 0.05 level (*p<0.05*) compared to PC. ^#^The mean difference is significant at the 0.05 level (*p<0.05*) compared to UC.

#### Evaluation of gastric protein concentration

The analysis of total protein revealed a significant (*p<0.05*) elevation of protein content to normal level in the ETHAB treated groups (Table 2). ETHAB (5 mg/kg) treatment resulted in an observed increase in total protein to 10.26±0.34 mg/mL as compared to the ulcer control group (7.28±0.51 mg/mL tissue). Increasing the ETHAB treatment resulted in a significant (*p<0.05*) increase in total protein content of 13.72±0.66 mg/mL of homogenate tissue (Table 2). Previously, a significant increase in total protein upon treatment with Schiff base Zinc II complex was reported in rats with acute superficial hemorrhagic mucosal lesions [6]. This observation was also found to be in accord with [13] on the gastroprotective potential of dichlorido-zinc(II) and dichlorido-copper (II) Schiff bases [44].

**Table 2:** Mean of total protein concentration, superoxide dismutase (SOD) activity and malondialdehyde (MDA) levels in stomach tissue homogenates of normal control, ulcer control, positive control, and ETHAB (5, 10 and 20 mg/kg) treated groups.

Animal Group	No of animals	Total protein (mg/mL tissue)	SOD (U/mg protein)	MDA (µmol/g protein)
**normal control**	6	12.17±0.37#	21.60±0.37* #	101.8±2.26#
**ulcer control**	6	7.28±0.51*	12.21±0.54*	204.2±3.77*
**positive control**	6	11.49±0.51#	28.81±1.33#	116.9±3.27#
**ETHAB (5 mg/kg)**	6	10.26±0.34*	18.29±0.51*	117.1±2.65#
**ETHAB (10 mg/kg)**	6	13.44±1.12#	23.36±0.79* #	124.04±5.35* #
**ETHAB (20 mg/kg)**	6	13.72±0.66#	25.55±1.12#	109.4±1.96#

*The mean difference is significant at the 0.05 level (*p<0.05*) compared to PC.

The article "Gastroprotective Activity of Ethyl-4-[(3,5-di-tert-butyl-2-hydroxybenzylidene) Amino]benzoate against Ethanol-Induced Gastric Mucosal Ulcer in Rats" was retracted in 2023. Reasons: duplicated images; overlap with earlier publications; original data or images not available; unreliable data.

# The mean difference is significant at the 0.05 level (*p<0.05*) compared to UC.

#### Antioxidant activity and MDA level in stomach homogenate

The superoxide dismutase (SOD) activity and malondialdehyde (MDA) level of each gastric sample were evaluated. One important function of SOD is the conversion of harmful superoxides to hydrogen peroxides, which are then converted to water molecules by catalase. Normally, in disease conditions, SOD level is observed to be highly reduced. In this study, SOD activity in the ulcer control group was also observed to be significantly (*p<0.05*) reduced. It is suggested that this reduction is likely to be due to the high utilization of SOD in the decomposition of superoxide anion generated by lipid peroxidation [12], [15], [45]. However, treatment with ETHAB increased SOD activity in a concentration dependent manner (Table 2). ETHAB treatment at a concentration of 5 mg/kg resulted in an observed increase in SOD activity of 18.29±0. U/mg protein. Increasing the concentration to 10 or 20 mg/kg resulted in a significant (*p<0.05*) increase in SOD activity (Table 2). Studies have shown a similar increase in SOD activity upon treatment with Schiff base complexes. Evaluating the gastro-protective potential of pre-treatment with Zinc II complexes, Golbabapour et al. [6] reported a significant (*p<0.05*) increase in SOD activity from 11.42±0.29 U/mg protein in the lesion control group to 24.96 U/mg protein in the 8.724×10^−5^ M/kg of Zinc II complex pre-treated group.

The lipid peroxidation assay evaluates the oxidative degradation of lipids, which causes disruption of cellular membranes. Cellular lipids that contain unsaturated fatty acids with more than one double bond are said to be more susceptible to the oxidizing action of free radicals [46], which leads to the generation of MDA as one of the major secondary oxidation products. In addition, MDA is reported to have mutagenic and cytotoxic effects [47]. In various diseases related to free radical damage, MDA level has been found to be elevated. Hence, it has been spectrophometrically used as a biomarker for the assessment of lipid peroxidation in the biological and medical sciences [47]. Schiff bases are reported to be cofactors for metallo-enzymes, superoxide dismutase (SOD), collagenase, alcohol dehydrogenase and spermatogenesis [13].

The article "Gastroprotective Activity of Ethyl-4-[(3,5-di-tert-butyl-2-hydroxybenzylidene) Amino]benzoate against Ethanol-Induced Gastric Mucosal Ulcer in Rats" was retracted in 2023. Reasons: duplicated images; overlap with earlier publications; original data or images not available; unreliable data.

The MDA analysis revealed the inhibition action of the compound on lipid peroxidation (Table 2). In comparison to the ulcer control group, ETHAB treatment of 5 mg/kg resulted in a significant (*p<0.05*) reduction of MDA level to 117.1±2.65 µmol/g tissue. On increasing the compound concentration to 20 mg/kg the MDA level was found to be further reduced to 109.4±1.96 µmol/g tissue. Similar studies have shown the reduction of MDA level upon treatment with Schiff bases and their complexes. Hajrezaie et al. [12] reported a significant (*p<0.05*) reduction of MDA level when 80 mg/kg of Schiff base derived from copper II complexes was used in evaluating gastro-protective effect. These results are also in agreement with reported MDA reduction during gastro-protection treatment with steroids [14], and Schiff base Zinc II complexes [6].

#### Gross appearance and histology of gastric mucosa

ETHAB pretreatment showed significant (*p<0.05*) reduction in the ulcerogenic area from 283.2±23 mm^2^ in the experimental group treated with 5 mg/kg to as low as 28.8±7 mm^2^ in the group treated with 20 mg/kg. This translates to an observed percentage in ulcer inhibition of 63.12 to 93.75% in groups treated with ETHAB (5 to 20 mg/kg), a value that is statistically similar to the observed percentage in ulcer inhibition (96.25%) in the positive control group (Figure 3c). This is in agreement with Golbabapour et al. [6], This observation is substantiated by the observed reduction of necrotic lesions in the hiostopathological micrographs (Figure 4c–f) upon treatment with either Omeperazole or ETHAB. In fact, the gross appearance of the necrotic lesions was observed to be significantly reduced upon ETHAB pretreatment in a concentration dependent manner. As shown in Figure 4d, pretreatment with 5 mg/kg ETHAB incurred a marked reduction of the hemorrhagic lesion when compared to the ulcer control group (Figure 4b). However, treatment with ETHAB 10 and 20 mg/kg resulted in a more prominent reduction of the lesion with visible flattening of the gastric mucosa (Figure 4e and f) to a level similar to that of the positive control group (Figure 4c). These observations are also found to be in agreement with previous literature [12], [13]. This effect could be due to the reported inhibition of leucocyte infiltration of the gastric wall in rats pretreated with ETHAB. It has been reported that up-regulation of COX-2 via COX-1 inhibition is the key factor in inflammatory reactions associated with ulcers [48]. Recently, Dwivedi et al. [49] demonstrated the possible role of Schiff bases in inhibiting inflammatory reactions by inhibiting the expression of the COX-2 enzyme. There have been similar reports on the inhibition of gastric mucosal lesions by hindering neutrophil infiltration in gastric ulcer tissue [50], [51]. The observed flattening of the gastric mucosa folds is said to be due to the relaxation of the circular muscles, which results in greater mucosal area exposure to the action of the pretreated compounds at the same time reducing the volume of gastric irritants on the regal crest [52].

The article "Gastroprotective Activity of Ethyl-4-[(3,5-di-tert-butyl-2-hydroxybenzylidene) Amino]benzoate against Ethanol-Induced Gastric Mucosal Ulcer in Rats" was retracted in 2023. Reasons: duplicated images; overlap with earlier publications; original data or images not available; unreliable data.

**Figure 4:** Gross lesion of the gastric mucosa in rats. (a) In rats pretreated with 10%Tween 20 without Eth-induced ulcer (normal control) no injury to the gastric mucosa appears. (b) Rats pretreated with 10% Tween 20 (ulcer control) followed with Eth-induced ulcer, have severe hemorrhage injuries in the gastric mucosa. (c) Rats pretreated with Omeprazole (20 mg/kg) have less injury to the gastric mucosa as compared to the ulcer control rats. (d) Rats pretreated with ETHAB (5 mg/kg) have moderate injuries in the gastric mucosa. The compound reduces the formation of gastric lesions induced by absolute ethanol. (e) Rats pretreated with ETHAB (10 mg/kg) have mild to moderate injuries in the gastric mucosa. (f) Rats pretreated with ETHAB (20 mg/kg) have mild lesions but significantly restored gastric mucosa with visible flattening of the mucosa.

Histopathological observation of the gastric lesions induced by orogastric intubation of ethanol revealed extensive damage in the ulcer control group (UC), corresponding to an ulcer area of 768±27 mm^2^ (Figure 3c). In comparison to the histological study of the stomach samples of the normal control group (Figure 4a), this observation is backed by the observed extensive black hemorrhagic lesions of gastric mucosa in the H&E stained micrographs of the ulcer control group in Figure 4b. Further histological observation of the sample's gastro mucosal cross-sections revealed the normal control group to have no signs of disruption to the gastric epithelium, submucosal edema or leucocyte infiltration (Figure 5a). It has been shown that feeding absolute ethanol extensively damages the mucosa and causes an increase of neutrophil infilteration into the mucosa in rats [22]. These infiltrated neutrophils are said to be the major source of inflammatory mediators, which results in the release of potent reactive oxygen species (ROS) that are highly cytotoxic and can interfere with the healing process of a gastric ulcer [22]. In contrast to Figure 5a, however, a severe disruption of the gastric mucosal epithelium lining in the ulcer control group was observed (Figure 5b). In this group, the necrotic lesions were observed to penetrate deeply into the mucosa (Figure 5b) with visible submucosal edema and extensive leucocyte infiltration. Experimental groups pretreated with either Omeprazole (Figure 5c) or ETHAB (Figure 5d–f), showed some mild edema and less superficial disruption of the gastric epithelial lining, with minor lesions of hemorrhagic necrosis. In fact, treatment with ETHAB at a higher concentration of 20 mg/kg (Figure 5f) resulted in comparatively better protection against the ethanol-induced gastric ulcer, due to a clear reduction of submucosal edema, leucocyte infiltration, with the epithelium lining being protected almost to the appearance of the normal control group. This observation is found to be in accord with similar reported observations on the gastro-protective effect of Schiff bases such as those of copper II complexes [44], Zinc II complexes [6] and indolic nickel II complexes [14].

The article "Gastroprotective Activity of Ethyl-4-[(3,5-di-tert-butyl-2-hydroxybenzylidene) Amino]benzoate against Ethanol-Induced Gastric Mucosal Ulcer in Rats" was retracted in 2023. Reasons: duplicated images; overlap with earlier publications; original data or images not available; unreliable data.

**Figure 5:** Histological study of ethanol-induced gastric mucosal damage in rats. (a) In rats pretreated with 10% Tween 20 (negative control) normal tissue has intact surface mucosal epithelium. (b). Rats pre-treated with 10% Tween 20 (ulcer control) have severe disruption of the surface epithelium and necrotic lesions that penetrate deeply into the mucosa (c) Rats pretreated with Omeprazole (20 mg/kg) have mild disruption of the surface epithelium mucosa, and there is a reduction in submucosal edema and leucocyte infiltration. (d) Rats pre-treated with ETHAB (5 mg/kg) have moderate disruption of the surface epithelium with edema and leucocyte infiltration of the submucosal layer. (e) Rats pretreated with ETHAB (10 mg/kg) have a mild to moderate disruption of the surface epithelium and a reduction in submucosal edema. (f) Rats pre-treated with ETHAB (20 mg/kg) have mild disruption of the surface epithelium (H&E staining; 10×).

#### Mucosal glycoprotein analysis

PAS of the mucosal glycoproteins revealed a noticeable increase in the level of PAS staining of gastric mucosa in the Omeprazole (Figure 6c) and ETHAB treated groups (Figure 6d–f) in comparison to the ulcer control group (Figure 6b). The observed intense magenta color in the apical epithelial cells of the treated groups indicated an increase in glycoprotein accumulation in the gastric mucosa. This intense coloration in the PAS staining photomicrograph was not observed in the ulcer control nor in the normal groups (Figure 6a), leading to less accumulation of glycoprotein. This observation is in agreement with previous observations [12]. The same sharp intense increase in magenta coloration of the glandular epithelial was also observed in the ulcer group pretreated with Schiff base Zinc II complex [6].

The article "Gastroprotective Activity of Ethyl-4-[(3,5-di-tert-butyl-2-hydroxybenzylidene) Amino]benzoate against Ethanol-Induced Gastric Mucosal Ulcer in Rats" was retracted in 2023. Reasons: duplicated images; overlap with earlier publications; original data or images not available; unreliable data.

**Figure 6:** Periodic Acid Schiff (PAS) staining of mucosal glycoproteins. The observed intense magenta color in the apical epithelial cells in the groups pretreated with ETHAB (d, e and f) and Omeprazole (c) compared with the ulcer control group (b) and normal group (a)(Magnification 10x).

#### Immunohistochemistry

Immunohistochemical analysis was observed based on the Hsp70 staining techniques as described in the methodology section. Hsp70 proteins are said to belong to a family of highly conserved universally expressed heat shock proteins having an approximate molecular weight of 70 kDa [53]. In fact, Hsp70 is reported to be among those proteins most abundantly produced in response to different cellular stresses in both prokaryotes and eukaryotes [54], [55]. This protein defends cells from oxidative stress and any injury-caused homeostatic process by acting as a molecular chaperone that inhibits proteins from aggregation, preserving the protein structure and allowing them to refold into their active conformation as well as repairing or removing damaged proteins [22], [55], [56]. Furthermore, these proteins are suggested to exert their cytoprotective function as cytokines via elucidation of their co-receptor CD14 [53].

Besides enhancement of gastric mucus secretion and the antioxidative capacity of these gastroprotective compounds, the mechanisms of action of these compounds have been speculated upon. Some researchers opine that the action is due to the modulation of inflammatory cytokine-mediated oxidative damage to the gastric mucosa [44], while others are of the opinion that the activity is due to the down regulation of the ulcer associated Bax protein with corresponding overexpression of the Hsp70 protein [22]. Studies have shown that the reactive oxygen species generated by the orogastric intubation of ethanol in rats suppresses the expression of Hsp70 proteins, while enhancing the over expression of Bax protein [6], [22]. In comparison to both normal control (Figure 7a) and ulcer control (Figure 7b) groups, the observed over-expression of Hsp70 proteins in both the positive control group (Figure 7c) and ETHAB pretreated groups (Figure 7d–f) could be sufficient for the gastro-protective efficacy of the compounds by up-regulation of Hsp70. Moreover, both the positive control group (Figure 8c) and ETHAB pretreated groups (Figure 8d–f) had remarkable down-expression of Bax protein in comparison to the ulcer group (Figure 8c), where the ethanol pretreatment up-regulated the expression of Bax. Golbabapour et al. [6] have shown that over expression of Hsp70 proteins is responsible for the gastroprotective action of Schiff bases of zinc II complexes. Similarly, AlRashdi et al. [22] have noted that over expression of Hsp70 and suppressed expression of Bax proteins could play an important role in protecting gastric mucosal damage. Consistent with previous literature [6], [22], [53], [56], this study has also shown that pretreatment with ETHAB results in a remarkably enhanced expression of Hsp70 protein and suppressed expression of Bax in the gastric mucosa of rats when compared to the ulcer control group. This demonstrates the cytoprotective function of Hsp70 and Bax protein once more.

The article "Gastroprotective Activity of Ethyl-4-[(3,5-di-tert-butyl-2-hydroxybenzylidene) Amino]benzoate against Ethanol-Induced Gastric Mucosal Ulcer in Rats" was retracted in 2023. Reasons: duplicated images; overlap with earlier publications; original data or images not available; unreliable data.

**Figure 7:** Immunohistochemistry staining of Hsp70 proteins. The analysis revealed an over expression of Hsp 70 protein in the stomach of rats pretreated with ETHAB(d, e and f) and Omeprazole (c) compared with the ulcer control group (b) and normal group (a)(Magnification 20x).

**Figure 8:** Immunohistochemistry staining of Bax proteins. The analysis revealed a down-expression of Bax protein in the stomach of rats pretreated with ETHAB (d, e and f) and Omeprazole (c) compared with the ulcer control group (b) and normal group (a)(Magnification 20x).

## Conclusions

Cytotoxic evaluation of the Schiff base ETHAB revealed that the compound exhibits the ability to proliferate the viability of WRL68, even at higher concentrations. The acute toxicity study showed that mice treated with the compound in concentration range of 500 to 1000 mg/kg show no mortality or any sign of toxicological complications. The antioxidant property of the compound was also ascertained by DPPH, FRAP, NO and metal chelating assays. In comparison to the negative control, treatment with the compound revealed increased protection of the gastric mucosa by increased gastric wall mucus, pH level of gastric contents and SOD activity, and a decrease in MDA level. It also produced a reduction in necrotic lesion, flattening of gastric mucosa, reduction of edema and leucocyte infiltration of the submucosal layer. There was an observed increase in PAS staining, up-regulation of Hsp70 protein and suppression of Bax protein expression. It is therefore concluded that Schiff base ETHAB has antioxidant and gastroprotective activity against ethanol-induced gastric ulcer.
